This article has been retracted.

# A Deep Learning and Clustering Extraction Mechanism for Recognizing the Actions of Athletes in Sports

**DOI:** 10.1155/2022/2663834

**Published:** 2022-03-24

**Authors:** Jianhua Yang

**Affiliations:** Anyang Institute of Technology, Anyang, Henan 455000, China

## Abstract

In sports, the essence of a complete technical action is a complete information structure pattern and the athlete's judgment of the action is actually the identification of the movement information structure pattern. Action recognition refers to the ability of the human brain to distinguish a perceived action from other actions and obtain predictive response information when it identifies and confirms it according to the constantly changing motion information on the field. Action recognition mainly includes two aspects: one is to obtain the required action information based on visual observation and the other is to judge the action based on the obtained action information, but the neuropsychological mechanism of this process is still unknown. In this paper, a new key frame extraction method based on the clustering algorithm and multifeature fusion is proposed for sports videos with complex content, many scenes, and rich actions. First, a variety of features are fused, and then, similarity measurement can be used to describe videos with complex content more completely and comprehensively; second, a clustering algorithm is used to cluster sports video sequences according to scenes, eliminating the need for shots in the case of many scenes. It is difficult and complicated to detect segmentation; third, extracting key frames according to the minimum motion standard can more accurately represent the video content with rich actions. At the same time, the clustering algorithm used in this paper is improved to enhance the offline computing efficiency of the key frame extraction system. Based on the analysis of the advantages and disadvantages of the classical convolutional neural network and recurrent neural network algorithms in deep learning, this paper proposes an improved convolutional network and optimization based on the recognition and analysis of human actions under complex scenes, complex actions, and fast motion compared to post-neural network and hybrid neural network algorithm. Experiments show that the algorithm achieves similar human observation of athletes' training execution and completion. Compared with other algorithms, it has been verified that it has very high learning rate and accuracy for the athlete's action recognition.

## 1. Introduction

With the continuous innovation of computer vision technology and the rapid development of multimedia and Internet technologies, people's ways of producing videos have gradually diversified and video resources have become more and more abundant. How to recognize human actions from videos has become a research direction of interest to people; the use of computer vision technology and rich video resources to identify human actions has become a research hotspot [1]. Action recognition based on video scenes uses computer vision, pattern recognition, machine learning, and other technical means to integrate video spatiotemporal feature information, detect one or more behavior segments, and classify them according to behavior categories [2]. The timing information of video can provide a lot of information for action recognition. How to make good use of the timing information in videos is the key to the research of action recognition algorithm [3].

In recent years, the research algorithms of action recognition are gradually developing, especially the action recognition algorithm based on deep learning, which greatly improves the accuracy of action recognition. From the recognition of simple actions in a single scene in the early stage to the recognition of complex actions in real natural scenes [4] and from the study of single-person action recognition to the study of interactive action and even large-scale group action recognition [5], this paper introduces three mainstream deep learning algorithm frameworks to solve the problem of motion recognition based on video spatiotemporal features: CNN-LSTM, 3D convolution, and dual stream network [6]. In addition, this paper will also briefly introduce the common databases of gymnastics teaching action recognition and the possible future development direction of action recognition algorithm based on deep learning [7].

Action recognition means that in gymnastics teaching, students can distinguish the perceived objects through various senses, proofread, and reject irrelevant stimuli, so as to obtain accurate action response information and master the action technology [8]. The ability of movement recognition is closely related to the existing sports knowledge and experience and has a direct impact on the formation process of movement skills and the teaching effect of gymnastics class [9]. Modern constructivism holds that although the world exists objectively, due to the different knowledge, experience, and social existence of each person, the understanding of the objective world and the judgment of things are different [10]. In the process of understanding and judging the objective world, there is bound to be a two-way and repeated interaction between external information and existing knowledge. The acquisition of new knowledge and the establishment of new experience are based on the existing knowledge and experience [11]. On this basis, modern constructivism gives a brand-new explanation to the modern teaching process, that is, in the teaching process, teachers should change from traditional knowledge transmitters to students' learning guides [12]. Students are builders of their own knowledge and the learning process is the process of constructing new knowledge [13]. In the learning process, based on the original experience system, students encode and combine new foreign information constantly and repeatedly, and the original knowledge and experience will be adjusted and enriched due to the entry of new information, thus constructing and forming new knowledge [14]. Using this viewpoint to reform the teaching mode of modern gymnastics and guide the teaching of modern gymnastics class is of great significance to cultivate students' learning enthusiasm, expand their knowledge, and improve their practical ability [15].

The rest of the paper is as follows: In Section 2, the related work is presented followed by the proposed work in Section 3. The experimental results are provided in Section 4. Finally, this paper is concluded and various research directions are provided in Section 5.

## 2. Related Work

Margarito et al. [16] found that the existing research results have good performance in dealing with short-term motion, but the performance of understanding long-term motion information is insufficient, and the training samples are small. Rothes [17] summarizes the application of machine learning in action recognition, and the system summarizes. The application of algorithms such as support vector machines and convolutional neural networks in computer vision is presented. Nagano et al. [18] recognized that the information obtained by the method of action classification after convolutional network and average prediction at the end is incomplete, especially in fine-grained action classification, it is easy to confuse action categories. Shurlock and Kelly [19] proposes a new convolutional neural network architecture and believes that the architecture can express a global-level description. The architecture adopts the method of temporal sharing parameters and optical flow in the implementation details. This method is used in the video classification task and shows excellent performance. The author proposes two methods for processing temporal information, one is feature pooling, that is, pooling through different positions. Briggs and Dreinhöfer [20] recognizes that for video action recognition, it is necessary to use higher-dimensional features to express the video, which in turn requires to collect more labeled data and do a lot of feature extraction. To avoid feature extraction work, one solution is to introduce unsupervised learning to discover and express video structure. Literature [21] proposes two LSTM models, which are called automatic encoder model and prediction model, respectively. The automatic encoder model inputs the frame sequence to the LSTM automatic encoder and then copies the representation vector learned by the LSTM automatic encoder to the LSTM decoder. The target sequence is the same sequence as the input, that is, reconstruct the image; the processing process of the prediction model follows the structure of the automatic encoder to predict the image. Finally, the author fused the two models. Literature [22] recognizes that the key to video analysis and processing lies in temporal features and the input and output of the network will become longer in the real scene. Therefore, the combination of LSTM and convolutional neural network can better learn spatial and temporal features. Literature [23] is limited to the shortage of data at that time. It decomposes the three-dimensional convolution into 2D spatial convolution and 1D temporal convolution, uses 2D convolution to learn video spatial features, and uses 1D convolution to learn temporal features. Compared with the three-dimensional convolution network, this network structure greatly reduces the amount of parameters and has low requirements for the amount of training data. The research in reference [24] further reveals the general processing process of pattern recognition. They believe that the recognition of surface and low-level features or the relationship between these features is the basis of judgment. The results show that the recognition performance of experts is better than novices in both video presentation and light spot presentation. Literature [25] puts forward the theory of long-term working memory, which holds that experts have developed complex task-related coding skills and are related to the retrieval structures in long-term memory. These retrieval structures enable experts to index and store information in the coding stage, such as features or the collection of features, allowing the upper-level representation of the current situation, which is conducive to the identification and prediction of events.

It can be seen from the literature that the ability of action recognition is closely related to the existing sports knowledge and experience, which has an important restrictive effect on the formation of action skills and directly affects the teaching effect of gymnastics classes. Therefore, teachers should constantly explore teaching laws, study teaching theories, improve teaching methods, activate classroom atmosphere, mobilize students' learning initiative, and cultivate students' ability to recognize movements, thereby promoting the formation of movement skills and improving the teaching effect of gymnastics classes.

## 3. Brief Description of the Method of Action Recognition Ability

### 3.1. Action Recognition on the Effect of Gymnastics Teaching

In gymnastics teaching, when teachers use movement demonstrations or picture demonstrations to show students a new movement, students first obtain information quickly through vision. Then, students will make preliminary judgments on the new movement based on the existing knowledge of the movement and form a hypothesis of “what is the current stimulus”, such as the body posture of the action, the height of the body's center of gravity, the body posture, the relationship between the body and the equipment, and the angle of the action; the information obtained visually enables the students to have a preliminary appearance impression of the newly learned action and make a plan for the ontology practice and corresponding preparatory responses. In addition, the accuracy of visual recognition will gradually improve with the accumulation of motor knowledge and the proficiency of motor skills. In gymnastics teaching, the teacher's demonstration of movements and teaching aids is not only the beginning of teaching activities, but more importantly, it enables students to directly obtain the appearance of movements through visual recognition. Therefore, according to different teaching tasks and the actual practice of students, it is particularly important to use targeted demonstrations and demonstrations. For example, complete movements should be accurate and standardized; partial movements should be clear and clear, induction exercises should be gradually migrated, key techniques should be highlighted, and the comparison between right and wrong should be rigorous and so on. Only in this way can students obtain accurate action information through visual recognition..

For the learning of any new action, while using action demonstration and picture demonstration, teachers should also explain the technology and principle of completing the action in detail and systematically and timely analyze and guide the students' practice. Such explanation and analysis is essential for students to further identify and understand movement technology. As one of the main channels to receive external information, the students' auditory system also plays a very important role in identifying information from teachers' language. This is because the information received by vision is only the appearance of action, while the information received by hearing is the deeper information of action, such as action structure, force sequence, key technology, and technical principle. It is worth noting that auditory recognition is not only closely related to students' existing knowledge and experience but also plays an important role in supplementing and strengthening the information obtained by previous visual recognition, which is helpful to a deeper understanding of action technology and speed up the formation of action skills. In teaching, in order to enable students to use the existing knowledge to quickly and accurately identify the language information from teachers, teachers are required to explain in a standardized and accurate way, with clear levels of action links, key technologies, concise and easy to understand language, and resolutely avoid ambiguous, ambiguous, and specious explanations.

The mastery of any new movement technique can only be achieved through constant physical exercises. Physical exercise is characterized by muscle activity, so it can be said that it is just empty talk to master the movement skills without muscle activity. The main features of muscle recognition are that only through repeated exercises and constant proofreading and correction can we gradually build up accurate proprioception of movement, such as the order of exertion, strength, posture of body, angle of movement, height change of center of gravity, relationship between body and instrument position, etc. The law of skill formation proves that the step-by-step induction exercise with a certain logical connection before and after has an important “transfer” effect on gradually establishing accurate proprioception of muscle movement, especially for movements with many technical links and relatively great difficulty. Using riding on the horizontal bar as the induction exercise on the front will help to realize the correct leg stretching direction, using goat full rotation as the transition exercise of pommel horse full rotation will help to establish the concept of umbrella full rotation, and using the handstand on the inverted frame as the auxiliary of parallel bars handstand. On the contrary, if the method adopted does not take into account the context of action links and the inherent law of muscle exertion, it will “interfere” with the establishment of proprioception of muscle movement. Therefore, according to this rule, teachers should adopt practical and effective teaching methods for different learning stages in teaching, so that students can speed up muscle identification and establish relevant technical concepts as soon as possible.

Brain recognition can also be called intuitive thinking; that is, the information of muscle activity appears in the brain in the form of kinesthetic images, and the brain makes judgments on the time, space, strength, and posture of the action and then readjusts and adjusts the muscle activity through the feedback loop. The movement will be made gradually accurate by corrections. The most important meaning of brain recognition is to analyze and process the incomplete and unsystematic information from the proprioception of muscles, constantly remove the false and preserve the true, remove the rough and extract the essence, from the outside to the inside, from here to there, so that the activities of the muscles gradually tend to be refined until the end. Build technical concepts. Teaching practice has proved that brain recognition has a remarkable feature. The first is that the speed of recognition is closely related to the flexibility of individual brain nerve cells, which is clearly manifested in the ability of muscle differentiation during movements; the second is that the accuracy of the feedback is restricted to a certain extent by the existing sports knowledge and skills. For example, the technology of raising the body's center of gravity and moving away from the rotation axis used in the first half of the front loop of the horizontal bar is based on the theory of biomechanics. The principle of the moment of gravity. The physics knowledge that students have mastered in middle school greatly promotes the speed of brain feedback, making movements more accurate and finer.

### 3.2. Action Recognition Framework Based on the Clustering Algorithm

The ability to perceive key information from complex environment plays an important role in successful operation in many fields of human activities. In the field of sports, this cognitive ability has been proved to be related to the recognition ability of athletes. Athletes can use this recognition ability to predict future events and guide their decisions and actions. Action recognition refers to the ability of the human brain to distinguish a perceived action from other actions and obtain predictive response information according to the changing motion information on the field. Motion recognition is a process of processing the relevant information of a specific sports situation with the help of the existing sports experience. The architecture of video database is shown in Figure 1.

The purpose of clustering analysis is to divide the objects in a set of objects into several small sets or categories, so that the objects in different classes are very different from each other, while the differences between the objects in the same class are very small. In cluster analysis, the label of each object is unknown, so cluster analysis is a method of unsupervised learning. Commonly used data types for cluster analysis are as follows: ① *Data Matrix*. The data matrix is also called the “object attribute” structure. For example, the object of planet can be characterized by attributes such as mass, radius, temperature, and rotation period. If there are *n* objects and each object has *m* features, the data matrix can be expressed as follows:

(1) $$\begin{array}{c} {\left(\begin{array}{cccc} x_{11} & x_{12} & \cdots & x_{1m}\\ x_{21} & x_{22} & \cdots & x_{2m}\\ x_{n1} & x_{n2} & \cdots & x_{\text{nm}} \end{array}\right)}_{n\times m}. \end{array}$$

The row of the second mock exam represents the object, the column represents the attributes of the object, and the entities represented by the row and column are different. ② *Similarity Matrix*. The similarity matrix, also known as the “object” structure, stores the similarity of all pairs of *n* objects, usually expressed as a *n* × *n* matrix:

(2) $$\begin{array}{c} \left(\begin{array}{cccc} s\left(1,1\right) & s\left(1,2\right) & \cdots & s\left(1,n\right)\\ s\left(2,1\right) & s\left(2,2\right) & \cdots & s\left(2,n\right)\\ \vdots & \vdots & \ddots & \vdots \\ s\left(n,1\right) & n\left(n,2\right) & \cdots & s\left(n,n\right) \end{array}\right), \end{array}$$

where *s*(*i*, *j*) represents the similarity between object *i* and object *j*. Both positive and negative values of *s*(*i*, *j*) can be taken. The greater the value of *s*(*i*, *j*), the more similar the two objects are. Generally, the similarity matrix is a symmetric matrix, namely, *s*(*i*, *j*)=*s*(*j*, *i*), but in some cases, the similarity matrix is also asymmetric. At this time, the similarity matrix does not meet the triangular law. The rows and columns of the similarity matrix represent the same entity, so the similarity matrix is called a single-mode matrix. The search engine establishes a connection between the video database and the user interface, extracts the features of query examples submitted by users, and matches them with the feature sets in the video index database. The architecture of the search engine is shown in Figure 2.

Typical clustering analysis methods mainly include the partition method, hierarchical method, density-based method, grid-based method, model-based clustering algorithm, model-based method, and constraint-based clustering. The video database includes video index database and original video file database. The index of video data is stored in the video index database; The original video file is stored in the original video file database. In this paper, scene description, key frame set, and key frame feature vector are used to construct the index of the original video file. In the scientific data analysis and engineering system, clustering data according to similarity measure is a key step. We use AP clustering algorithm (Affinity Propagation clustering algorithm) to cluster video sequences. The AP clustering algorithm is derived by applying the max-product algorithm on a weighted graph, and it clusters according to the similarity between *n* data points, which make up the similarity matrix *S*(*i*, *k*) of *n* × *n*. The similarity *S*(*i*, *k*) indicates the suitability of the point of data point *k* as the cluster center of data point *i*. In general, the similarity can be set as the Euclidean distance. For point *x*_*i*_ and point *x*_*k*_, the similarity can be defined as follows:

(3) $$\begin{array}{c} s\left(i,k\right)=-{\left\|x_{i}-x_{k}\right\|}^{2}. \end{array}$$

The clustering results can be evaluated by calculating the net similarity. Net similarity is defined as the sum of the sum of noncentral data points and their respective central data points and the sum of their own reference degrees. Its formula is as follows:

(4) $$\begin{array}{c} \text{net similarity}=\sum_{k=1}^{k}\sum_{i=1}^{i_{k}}s\left(i,k\right)+\sum_{k=1}^{k}p\left(k\right). \end{array}$$

The larger the net similarity value, the better the clustering result.

The cyclic neural network algorithm uses the input sequence, output sequence, and hidden sequence, in which the historical records of the input sequence are also saved. The cyclic network is used to transfer the preceding item, and the transfer formulas are as follows:

(5) $$\begin{array}{c} h_{t}=\text{sigmoid}\left(W_{{\text{xhX}}_{t}}+W_{{\text{hhh}}_{t-1}}+\text{Ch}\right), \end{array}$$

(6) $$\begin{array}{c} z_{t}=\text{sigmoid}\left(\text{Whzht}+\text{Cz}\right). \end{array}$$

Finally, obtain the output result value of the next layer as shown in

(7) $$\begin{array}{c} \text{Ot}=\text{sigmoid}\left[\text{Wo}\left(h_{t-1}x_{t}\right)+c_{o}\right]. \end{array}$$

In the forget gate formula, AA is used to identify the output result of the previous round, and BB represents the current data conclusion. The main function of the user interface is to provide users with various query methods, including video input, image instance input, template input, or keyword input, to support users to choose convenient query methods in different application scenarios. The user interface architecture is shown in Figure 3.

To sum up, it can be seen that the fourth-layer clustering algorithm in the multilayer hybrid clustering algorithm takes the feature centers output by the third-layer clustering algorithm as input, uses the DBSCAN algorithm for clustering, and extracts the class centers as the multilayer clustering algorithm. The subactions common to each main action, in which the outliers are used as action features alone, and the feature centers of different main actions are determined according to the outliers in different data sets. The normalized value of the distance is used to judge the probability of the action occurring.

## 4. Result Analysis and Discussion

With the continuous improvement of people's quality of life, people will follow various standard fitness videos to exercise, but because there is no on-site guidance from professional coaches, the body is often injured due to nonstandard movements, ranging from muscle strain to severe fractures. Therefore, it is necessary to identify whether the movements of sports are standard, and to discover nonstandard movements in time, and then correct them. The existing recognition methods are roughly divided into two types: one is for image recognition, which has the advantage of being accurate, but the disadvantage is that it cannot be processed for a video, and the real-time performance is poor; the other is for video recognition, but most of them are for each frame. Compared with the standard image, the advantage is that the image can be processed in real time. The invention aims to solve the above technical problems existing in the prior art and provides a real-time and accurate sports video action recognition method based on action hotspot map. The parameter value setting of convolution kernel plays a key role in the classification and recognition results. If its value is small, the identification ability of the classified pictures to be extracted will be reduced, its value is large, large picture noise will be generated, unnecessary classification will be increased, and the requirements of calculation and storage capacity will also be raised. At the same time, the convolution kernel itself is subject to the dual effect of space-time dimension. Combined with the previous research results and the experiments of three-dimensional deep convolution neural network structure and athlete's action recognition and judgment for many times, it is found that the neural network structure with convolution kernel as the 4 *∗* 4 *∗* 4 matrix has the best effect. (Convolution kernel size 3 *∗* 3 *∗* 3, 4 *∗* 4 *∗* 4, 5 *∗* 5 *∗* 5.) The comparison of motion recognition segmentation accuracy of convolution kernels with different sizes is shown in Figure 4.

The pooling kernel of the convolution algorithm is related to the convolution kernel. The function of the pooling kernel is to reduce the dimension of the feature map, improve the resolution ability, and reduce the probability of image fitting in advance. The size of the convolution kernel determines the dimension of the pooling kernel. If the pooling kernel is too large, the action information will be filtered out. If the pooling kernel is too small, the pooling task cannot be completed. Combined with the previous research, the algorithm in this paper selects a 3 *∗* 3 *∗* 3 matrix as the pool. Nucleus. The test process is mainly to perform model training on action pictures and perform a large number of iterative training on optical flow data and RGB image data, respectively. The action recognition accuracy of the two variables is positively correlated with the number of trainings which is shown in Figure 4. The optical flow data and the number of neural network loops increase greatly before 15,000, but the accuracy comes to be stable in that region later. The critical threshold of the RGB airborne network is smaller, it stabilizes after 9000 cycles, and the accuracy of both is above 95%. RGB refers to three-color primary light image data. The RGB color mode is a color standard in the industry. It obtains various colors by changing the three-color channels of red (R), green (G), and blue (B) and superimposing on each other. RGB is the color representing the three channels of red, green, and blue. This standard includes almost all colors that can be perceived by human vision and is one of the most widely used color systems at present. The comparison of RGB and optical flow graph training accuracy is shown in Figure 5.

The performance of the AP clustering algorithm is mainly influenced by two parameters: reference degree and damping coefficient. The reference degree indicates the similarity between a data point and itself, and the number of categories finally obtained by clustering is influenced by it. On the other hand, the AP clustering algorithm often leads to the oscillation of iterative process due to the overshoot of the results in the iterative calculation process because the damping coefficient needs to be added to prevent this from happening. The influence of the damping coefficient *λ* on the iterative process is shown in Figure 6.

It can be seen from Figure 6 that the number of iterations increases with the increase of damping coefficient *λ*, and when there are many clustering data points, very small damping coefficient *λ* will make the iterative process difficult to converge. However, the jitter of the objective function, that is, the net similarity value, will decrease with the increase of the damping coefficient *λ* in the iterative process, thus ensuring the convergence of the iterative process at the cost of increasing the number of iterations. The performance comparison between AP algorithm and APLS algorithm is shown in Figure 7.

In order to further verify that the clustering motion combination method proposed in this paper has a good effect on the key frame set extracted from different video types, especially for video types with many scenes, complex content, and intense motion, this method is compared with several typical video key frame extraction methods. This paper makes analysis and comparison from two angles: first, when the clustering algorithm is also used, the multi-feature fusion measure in this paper is compared with the single feature measure of other clustering based methods; The second is to compare the proposed method with other types of key frame extraction methods. The comparison of clustering based method is carried out with sampling-based method and shot-based method. From the fidelity contrast curve, we can draw the following conclusions: for the video with more intense action and greater scene change, the quality of the extracted key frames is better than other methods. The fidelity contrast curve of sports video is shown in Figure 8.

It can be seen from the fidelity comparison curve that for videos with violent motion and rapid scene changes, the set of key frames extracted by a single feature description is not enough to represent the original video sequence. For the changed video category, the experimental effect of using a single feature description is not much different from the experimental effect of multifeature fusion. The comparison curve of sports video compression rate is shown in Figure 9.

From the compression ratio comparison curve, the following conclusions can be drawn: Because the strategy for selecting key frames in this paper is to select the frame at the minimum value of motion as the key frame in the interval with a specific length, the compression ratio is insensitive to the video type. For shot-based methods, the higher the number of shots, the more complex the motion and the worse the compression. For the sampling-based method, the compression ratio is insensitive to the video type, the higher the compression ratio, the lower the fidelity; the lower the compression ratio, the higher the fidelity. For video types with complex content, numerous scenes, and rich actions, the method proposed in this paper ensures high fidelity while ensuring a high compression rate.

To sum up, when compared with several classical algorithms, because the algorithm proposed in this paper introduces feature normalization processing and multiframe data recognition and processing, the accuracy of data recognition and execution are improved significantly better than other algorithms in time.

## 5. Conclusions

By summarizing the research progress of athletes' technical and tactical pattern recognition characteristics and cognitive neural mechanism, it is not difficult to find that the research on sports technical action pattern recognition is still in progress due to its implicitness or limitations of research methods. It cannot be in-depth, but the pattern recognition is a key link in sports technical judgment and decision-making. Before accurate prediction or successful decision-making, athletes must first identify the sports situation or sports technology. Specifically, the pattern recognition process is used to judge the outcome of the motion context and to determine whether the current context has been seen before, including the process of encoding and characterizing similar target cues. Another theory holds that recognition skills are only a byproduct of the cognitive processing of specific tasks and act as a reasonable indicator of the knowledge structure mastered by individuals and are not directly related to predictive skills. Therefore, it is imperative and significant to develop scientifically effective research methods and experimental paradigms to deeply explore them. By summarizing the research progress of athletes' technical and tactical pattern recognition characteristics and cognitive neural mechanism, it is not difficult to find that due to the implication or limitations of research methods, the research on sports technical action pattern recognition is still in progress. Pattern recognition is a key link in motion technology judgment and decision making. Before accurate prediction or successful decision making, athletes must first determine the sports situation or sports technology. Specifically, the pattern recognition process is used to judge the result of the motion context and determine whether the current context has been seen before, including the process of encoding and describing similar target clues. Another theory holds that cognitive skills are only the byproduct of the cognitive process of specific tasks. They are a reasonable index for individuals to master the knowledge structure and have no direct relationship with prediction skills. Therefore, it is of great significance to develop scientific and effective research methods and experimental paradigms. In recent years, researchers in various countries have made a lot of progress in the field of action recognition, and the test results of public datasets in international competitions have also been greatly improved. In the future, action recognition methods based on deep learning will also have more in the following aspects. Development: (i) Extract multimodal and multifaceted features. Multimodality and multifeatures can give more information to deep neural networks, and the fusion of multiple features must be the direction of future development, such as combining audio and video features for action recognition. (ii) Build large-scale general data sets. Action recognition has been able to achieve high accuracy on various existing data sets, and the construction of larger scale, more scenes, and more abundant action composition general data sets is closer to practical application scenarios. (iii) Improve algorithm efficiency and classification accuracy. With the continuous improvement of the real-time requirements of the algorithm, improving the detection speed of the action recognition deep learning framework will also be the future development direction. At the same time, research on fine-grained action recognition with subtle changes will also attract much attention.

## Figures and Tables

**Figure 1:** Video database architecture diagram.

**Figure 2:** Retrieval engine architecture diagram.

**Figure 3:** User interface architecture diagram.

**Figure 4:** Comparison of motion recognition segmentation accuracy of convolution kernels with different sizes.

**Figure 5:** Comparison of training accuracy between RGB and optical flow diagram.

**Figure 6:** Influence of the damping coefficient *λ* on the iterative process.

**Figure 7:** Performance comparison between AP algorithm and APLS algorithm.

**Figure 8:** Sports video class fidelity comparison curve.

**Figure 9:** Comparison curve of sports video compression ratio.

## Data Availability

All the data used to support the findings of this study are included in the paper.
